# Angelica sinensis polysaccharide prevents mitochondrial apoptosis by regulating the Treg/Th17 ratio in aplastic anemia

This article has been retracted.

**DOI:** 10.1186/s12906-020-02995-4

**Published:** 2020-06-22

**Authors:** Zetao Chen, Li Cheng, Jing Zhang, Xing Cui

**Affiliations:** 1 Department of Gerontology, Affiliated Hospital of Shandong University of Traditional Chinese Medicine, Jinan, 250014 China; 2 Department of Acupuncture, Affiliated Hospital of Shandong University of Traditional Chinese Medicine, Jinan, 250014 China; 3 Department of Science and education, Shandong Mental Health Center, Jinan, 250014 China; 4 Department of Hematology, Affiliated Hospital of Shandong University of Traditional Chinese Medicine, 16369 Jingshi Road, Jinan, 250014 China

**Keywords:** Aplastic anemia, Mitochondria, Apoptosis, Treg, Th17, P38/MAPK

## Abstract

**Background:**

Angelica sinensis polysaccharide (ASP) is an effective medicine for aplastic anemia (AA). The present study aims to investigate whether mitochondrial apoptosis in aplastic anemia could be corrected by ASP by adjusting an abnormal level of regulatory T cell (Treg)/ IL-17 secreting CD4 T cell (Th17) ratio.

**Methods:**

BALB/c mice were treated with 5.0 Gy Co60 γ -radiation. Then 2 × 10^6^ lymph node cells from DBA/2 donor mice were transplanted within 4 h after radiation. The mice in the various groups were fed saline or ASP for 2 weeks. For the in vitro experiment, bone marrow nucleated cells (BMNCs) and Treg cells were sorted from the mice on the 2nd day of modeling, and then cultured with or without ASP.

**Results:**

The mice treated with the medium dose of ASP for 14 days showed increased white blood cell (WBC), red blood cell (RBC), platelet (PLT), BMNC counts and Lin–Sca-1 + c-Kit+ (LSK) populations viability compared with the mice in the AA group mice. The data showed that ASP decreased damage to the mitochondrial outer membrane, improved the stabilization of the mitochondrial membrane, and corrected the abnormal levels of ROS and mitochondrial-associated apoptosis proteins, including the Bcl-2/Bax ratio and caspase-3 and caspase-9 expression, in BMNCs which were sorted from the bone marrow cells of AA mice. The changes to the p-P38/P38 and Treg/Th17 ratios induced by AA were also reversed by the medium dose of ASP. The same ASP effect including the Bcl-2/Bax and p-P38/P38 ratio, caspase-3 and caspase-9 expression of BMNCs were observed in vivo. The viability of Treg cells were increased by treatment of ASP in vivo.

**Conclusions:**

ASP might prevent mitochondrial apoptosis to restore the function of hematopoietic stem cells by suppressing abnormal T-cell immunity in AA.

## Background

Aplastic anemia (AA) is considered a bone marrow failure syndrome because it is characterized by peripheral pancytopenia and marrow hypoplasia. Several studies have confirmed that T helper (Th) cells, such as IL-17-producing (Th17) CD4+ T cells, play a negative role in the pathogenesis of AA [1], whereas regulatory T cells (Tregs) maintain immunological self-tolerance and immunosuppression [2], which play a critical role in protection of the hematopoietic function in AA [3]. However, whether mitochondrial apoptosis influences hematopoietic stem cells in AA remains unknown.

Mitochondria are described as the “energy factory of a cell” because they produce adenosine triphosphate (ATP) [4]. Additionally, mitochondrial DNA (mtDNA) has a very high mutation rate due to the lack of protective histones and an effective DNA repair system. Mutations in mtDNA are associated with hematological diseases, such as acquired sideroblastic anemia, myelodysplastic syndromes and acquired AA [5–7]. Our previous study [8] showed that mutation-induced functional impairments of the mitochondrial respiratory chain might be involved in hematopoietic failure in AA patients. Abnormal mitochondrial membrane permeabilization and the morphological features of end-stage cell death (apoptotic, necrotic, autophagic, or mitotic death) are characteristic factors in not only the survival but also the death of cells [9].

*Angelica sinensis*, the most important herb in Dang-Gui-Bu-Xue decoction, could increase the quantity of red blood cells (RBCs), white blood cells (WBCs) and bone marrow nucleated cells (BMNCs), promote the proliferation of BMNCs and increase the quantity of multilineage progenitor cells (CFU-Mix) in a mouse model [10]. Previous studies have also shown that *Angelica sinensis* polysaccharide (ASP) can protect the hematopoietic function of CD34+ cells against adriblastin [11], improve the hematopoietic function of CD34+ hematopoietic stem/progenitor cells (HSPCs) by mitigating oxidative damage to stromal cells [12], and protect against X-ray irradiation-induced aging by inhibiting oxidative stress damage [13]. In addition, ASP promotes hematopoiesis and thrombopoiesis through the PI3K/AKT pathway [14]. We also confirmed the effect of ASP on mitochondrial membrane stabilization in another AA model by evaluating the number of mitochondrial, and concentration time curves of COX and MDH [15]. However, the anti-apoptotic function of ASP remains unknown.

The purpose of this study was to investigate whether ASP can effectively treat the hematopoietic stem cells (HSCs) of AA mice through the mitochondrial apoptosis signaling pathway regulated by Treg cells.

## Methods

### Materials

ASP with > 98% purity was purchased from Ci Yuan Biotechnology Co., Ltd. Shanxi (Xian, China). Dimethyl sulfoxide (DMSO), trypsin, 2′,7′-dichlorofluorescin diacetate (DCFH-DA), and PrestoBlue™ Cell Viability Reagent were purchased from Thermo Fisher Scientific (Shanghai, China). The 5,5′,6,6′-tetrachloro-1,1′,3,3′-tetra-ethylbenzimidazolcarbocyanine iodide (JC-1) assay kit, Annexin V-FITC/PI kit, and protein extraction and quantitation kits were purchased from Nanjing Jiancheng Bioengineering Institute (Nanjing, China). Cleaved caspase-9, cleaved caspase-3, Bax, Bcl-2, p-p38, and p38 were purchased from Cell Signaling Technology. β-actin was purchased from Abcam Co. FITC-labeled antibodies against lineage markers, including macrophage-1 antigen (Mac-1), Gr-1, Ter119, CD4, CD8a, CD3, B220, c-Kit-APC and Sca-1-PE, were purchased from BD Biosciences (Shanghai, China). A mitochondria isolation kit was purchased from Beyotime Biotechnology Inc. (Beijing, China). A functional mitochondria isolation kit, mitochondrial outer membrane integrity testing kit, mitochondrial inner membrane integrity testing kit, purified mitochondrial cytochrome C oxidase activity assay kit, reactive oxygen species (ROS) assay kit and phosphate-buffered saline (PBS) were obtained from Wuhan Boster Biotechnology, Ltd. (Wuhan, China). The cell lysis buffer and horseradish peroxidase-conjugated secondary antibodies used for Western blotting were obtained from Beyotime Biotechnology (Shanghai, China).

### Induction of AA and drug treatment

Sixty-four Healthy male BALB/c mice (weighing 18–22 g and aged 6–8 weeks) were provided by the Experimental Animal Center of Shandong University (China). The animals were housed in a warm, quiet environment with free access to food and water and acclimatized for 1 week prior to the initiation of the experiments.

The 64 mice were randomly divided into groups: the negative control group,the normal control group (low-dose group, medium-dose group and high-dose group, the data was showed in supplementary Fig. 2), the model group and three treated groups (low-dose group, medium-dose group and high-dose group). The AA model was established as previously described [16]. Briefly, the mice were irradiated with 5.0 Gy Co60 γ-radiation,then 2 × 10^6^ lymph node cells from DBA/2 donor mice were transplanted within 4 h after radiation (Fig. 1a).

**Fig. 1:** Assessment of the establishment of the AA model in the normal and model control groups based on the peripheral blood cell and BMNC counts (x ± SD) and bone marrow biopsies. **a**: Detailed experimental flow of the animal handling. **b**: Peripheral blood cell and BMNC counts in the different groups. **c**: Bone marrow biopsy of the normal group, model control group and different dose ASP groups on day 14. As indicated by the arrows,we can observe that hematopoietic tissue was replaced by adipose tissue in the AA model groups. The hematopoietic area in the treated group was appreciably larger than that in the AA group. **d**: The mitochondrial structure was detected by electron microscopy (× 16,500) on day 14. As indicated by the arrows, destroyed mitochondria were detected. Note: ▲*P* < 0.05 and ▲▲*P* < 0.01 compared with the normal control group. *P < 0.05 and **P < 0.01 compared with the model control group; #*P* < 0.05 and ##*P* < 0.01 compared with the low-dose group

The normal control group and treated group was intragastrically fed ASP (100, 200, and 400 mg/kg/d, according to the Chinese Medical Dictionary, Mu’s study [13] and our data). For the acute or chronic toxicity test, the maximum tolerated dose (2400 mg/kg/d) of ASP was used for 2 or 14 consecutive days, respectively. These data are shown in supplementary Fig. 1, which showed no toxicity of ASP in mice. The mice in the normal control and model groups were intragastrically fed a diet supplemented with physiological saline (10 ml/kg/d). In addition, all the mice received a standard diet throughout the study. After treatment with ASP or physiological saline for 2 weeks, euthanasia was performed by cervical dislocation on day 14. Before euthanasia, blood was collected by puncturing the caudal vein and after the animals were killed by cervical dislocation, the femur and spleen were removed immediately. Four mice in the AA group died during the first week, and two mice in the treated groups died within the first 2 weeks.

### Peripheral blood BMNC counts and bone marrow biopsy examination of mice

Tail vein blood samples were collected from the mice in all the groups on day 14. WBCs, RBCs and PLTs were counted in the peripheral blood samples. At the end of the experimental period, the mice were sacrificed AND met euthanasia criteria, and femur smears were prepared to performdifferential counting of BMNCs and bone marrow biopsy.

### Analysis of the cell viability of Lin^−^Sca-1^+^c-kit^+^ (LSK) populations

The bone marrow cells from the animals in the AA groups were obtained on day 14. For sorting of hematopoietic stem and progenitor cells, Lineage negative cells were harvested by MACS according to protocol of a mouse lineage depletion kit (Miltenyi Biotec, Italy), followed by sorting for HSPCs and HSCs (LSK, and LSKCD34 markers) with FACS (BD Ari III, USA). The subsequent HSPCs or HSCs cells were either analyzed with flow cytometry or transiently cultured in IMDM containing 20% FBS (Hyclon, USA), IL-6, Flt-3, SCF, IL-11 (PeproTech, Rocky Hill, USA). The viability of LSKs was assessed using the Presto Blue Assay with 96-well black plates. After 4 μl of PrestoBlue reagent was added to the 96 black plates, the plate was incubated for 30–45 min at 37 °C in an incubator, and the fluorescence was then measured using a Biotek plate reader. After background subtraction, the fluorescence of the sample was divided by the highest fluorescence in the row.

### Flow cytometric analysis of surface receptor expression in the spleen

The mAbs for mouse CD3-FITC, CD4-FITC, CD8-PE, CD25-PE, Foxp3-PE-Cy5 and IL-17-PE were purchased from BD Biosciences (USA), and the fixation/permeabilization reagent kit was purchased from Beckman Instruments, Inc. The cells were incubated with antibodies on ice for 30 min, washed twice with phosphate buffered saline (PBS), and resuspended, and their phenotypes were detected through flow cytometric analysis using the FACSCalibur flow cytometer (BD Biosciences). When testing Foxp3, single cell suspensions from the spleen were stimulated with PMA & Ionomycin for 4 h. The ratio of Treg cells to Th17 cells was calculated.

### Analysis of apoptosis and ROS

Cell apoptosis of BMNC cells cultured for 48 h was quantified using an Annexin V-FITC kit according to the manufacturer’s instructions and analyzed by flow cytometry (BD Biosciences, San Jose, CA, USA). The specific probe DCFH-DA was used to determine the content of intracellular ROS in BMNC cells according to the manufacturer’s instructions. Photographs of the cells were taken using an inverted fluorescence microscope (Olympus, Osaka, Japan).

### Assessment of mitochondrial outer membrane integrity

Mitochondria were extracted from BMNCs at 0 h, 24 h, 48 h, and 72 h using a high-purity mitochondrial isolation kit, and the total mitochondrial protein was quantified using the Coomassie brilliant blue method. The mitochondrial samples were tested according to the instructions of the UENMED Mito Outer Membrane Integrity Testing Kit using a spectrophotometer at a wavelength of 550 nm. The percentage of damage to the mitochondrial outer membrane was calculated based on the cytochrome oxidase (COX) levels using the following formula: COX level in diluent/total COX level in the lysis buffer.

### Assessment of mitochondrial inner membrane function

To detect variations in the mitochondrial membrane potential (MMP, ΔΨm) in the BMNCs, we used flow cytometry combined with JC-1 staining.

Isolated cells (0.5 × 10^6^ cells) were resuspended in 0.5 ml of PBS, and 500 μl of JC-1 working solution was added to the cells. The cells were then incubated at 37 °C in 5% CO_2_ for 15 min, centrifuged and resuspended in JC-1 working solution. The changes in the levels of red and green fluorescence were detected by flow cytometry.

### BMNCs for in vitro experiments

For the in vitro experiments, BMNCs were obtained from normal or model mice at d2. After that, samples from the control group were cultured in IMDM (Thermo Fisher Scientific) supplemented with 10% FBS (Biological Industries, Beit-Haemek, Israel) and antibiotics (100 u/ml penicillin and streptomycin). The treated group was cultured in the same medium supplemented with FBS and antibiotics and containing ASP (100,200 and 400 ng/ml were chosen according to our preliminary data). These cells were cultured in a humidified incubator containing 5% CO_2_ at 37 °C and were tested for viability and apoptosis proteins levels at 0 h, 24 h and 48 h.

### Treg cells for in vitro experiments

For the in vitro experiments, Treg cells were sorted from the spleens of normal or control model mice by using a BD FACSAria II at d2. We used FITC-labeled antibodies against lineage markers, including CD8、CD25 and CD127 antibodies. Then, samples from the control group were cultured in IMDM (Thermo Fisher Scientific) supplemented with IL-2, TGF-βand 10% FBS (Biological Industries, Beit-Haemek, Israel) and antibiotics (100 u/ml penicillin and streptomycin). Samples from the treated group were cultured in the same medium containing ASP (100,200 and 400 ng/ml). These cells were cultured in a humidified incubator containing 5% CO_2_ at 37 °C and were tested for viability at 0 h, 24 h and 48 h.

### Western blot analysis

BMNCs were lysed using a cell lysis buffer for Western blotting, and 40 μg of protein from each sample was separated on a 12% SDS-PAGE gel. The proteins were then transferred electrophoretically to 0.45-μm nitrocellulose membranes, and the membranes were incubated overnight with primary antibodies against Bcl-2, Bax, p38 and β-actin levels at 4 °C and then with secondary antibodies. The band intensities were quantified using ImageJ software (National Institutes of Health, Bethesda, MD, USA).

### Statistical analysis

The statistical analyses were performed using SPSS 19.0 software, and the data are expressed as the means±SDs. One-way ANOVA was used to test the differences among groups, and Scheffe’s modified F-test was subsequently used for multiple comparisons. A value of *P* < 0.05 was considered to indicate statistical significance.

## Results

### Effects of ASP treatment on enhancing peripheral blood cells, BMNC counts and the hematopoietic tissue area in bone marrow biopsies from AA mice

Using a fully automated blood cell analyzer, we found that the numbers of peripheral blood cells and BMNCs and the hematopoietic tissue area in bone marrow biopsies from the AA mice were notably decreased (*P* < 0.05), which indicated successful establishment of the AA mouse model (Fig. 1b-c). Significant destroyed structures of mitochondria including an absent ridge and mitochondrial swelling were observed in the AA model control group and low dose ASP group (Fig. 1d). After these mice were treated with ASP for 14 days, the WBC/RBC/PLT and BMNC counts were increased compared with those in the model group (*P* < 0.05 or *P* < 0.01; Fig. 1b), but the hematopoietic tissue area in the bone marrow biopsies showed no significant differences among the three treated groups. The WBC/RBC/PLT and BMNC counts were also detected in normal mice after treatment with different doses of ASP, as shown in supplementary Fig. 2, there was no significant difference between these groups and the normal blank group.

### Cell count and viability of LSKs

After LSK cells were obtained from bone marrow, the cell count and viability of LSK cells were tested. The first important finding was the high degree of reduction, even though hardly any cells were obtained from the AA group after 48 h. After treatment with medium dose of ASP, the level of LSK cells was recovered significantly compared with the other treatment group (Fig. 2a). The PrestoBlue Assay was adopted to measure the cell viability of LSKs. As shown in Fig. 2b, the viability of the LSK cells in AA mice was significantly lower than that in the normal controls.

**Fig. 2:** Effect of ASP on the number of LSK cells and the Treg/Th17 ratio. **a**: The number of LSK cells of different AA groups was detected to assess the efficacy of ASP. **b**: The cell viability of LSK cells was detected by PrestoBlue Assay. **c**: The Treg/Th17 ratio in different AA groups. **d**: Treg cells were detected by FCM. E: Th17 cells were detected by FCM. Note: ▲*P* < 0.05 and ▲▲*P* < 0.01 compared with the normal control group. *P < 0.05 and **P < 0.01 compared with the model control group; #*P* < 0.05 and ##*P* < 0.01 compared with the low-dose group; ■*P* < 0.05 compared with the medium-dose group

### Regulation of the abnormal Treg/Th17 ratio through treatment with ASP

CD4 + CD25 + FOXP3+ Tregs are indispensable for the maintenance of immunological self-tolerance and immunosuppression [17, 18], and impaired Treg function has been associated with AA pathogenesis [19]. As shown in Fig. 2c-e, the Treg/Th17 ratio in the AA mice recovered after ASP treatment.

### Mitochondrial ultrastructure of BMNCs

Mitochondrial apoptotic features, which are characterized by abnormal chromatin condensation on the nuclear membrane, mitochondrial swelling, and cristae breakage, were detected in BMNCs (Fig. 1d). Mitochondrial apoptotic features, which include abnormal chromatin condensation on the nuclear membrane, mitochondrial swelling, and cristae breakage, were enhanced after treatment with 200 mg/kg/d ASP (Fig. 1d).

### Effects of ASP on ROS and apoptosis

To study the induction of apoptosis, we examined the BMNCs from the different groups. As shown in Fig. 3a and e, ASP treatment decreased the cell apoptosis ratio compared with that of the model control group (30.23 ± 5.36). A clear significant decrease in the cell apoptosis ratio was observed (*P* < 0.01), and the best effect was obtained with the medium dose (Fig. 3a, e).

**Fig. 3:** Effects of ASP on mitochondrial apoptosis in LSK cells. **a**: Apoptosis was assessed in different groups. **b**: The ROS levels were assessed by inverted fluorescence microscopy. **c**: The MMP levels were tested by using flow cytometry. **d**: Outer membrane integrity was assessed. E: Flow cytometry scatter plot of apoptosis. **f**: Immunofluorescence images of ROS. G: Flow cytometry scatter plot of MMP. **h**, **i**: Markers of mitochondrial apoptosis and the p38/MAPK signaling pathway were tested by Western blotting. The results for the treated group indicate that the medium-dose ASP treatment reduces mitochondrial apoptosis in BMNC cells. Note: ▲*P* < 0.05 and ▲▲*P* < 0.01 compared with the normal control group. *P < 0.05 and **P < 0.01 compared with the model control group; #*P* < 0.05 and ##*P* < 0.01 compared with the low-dose group; ■*P* < 0.05 compared with the medium-dose group

The mean fluorescence intensity of ROS was quantified (Fig. 3b, f), and the results showed that ASP at a concentration of 200 mg/kg/d significantly decreased intracellular ROS levels compared with the model control group.

### Induction of mitochondrial signaling pathway by ASP treatment

MMP is an important parameter of mitochondrial function, and the collapse of the MMP was assessed by JC-1 staining. We analyzed the fluorescence ratio from flow cytometry data based on the progressive efflux of JC-1 from the mitochondria to the cytoplasm, which signaled disruption of the MMP (ΔΨm). The results showed that the MMP in bone marrow cells from the medium-dose group (8.30 ± 2.30) was significantly higher than that in the cells from the model control group (1.19 ± 0.77) (*P* < 0.01) (Fig. 3c, g), which indicated a loss of MMP during apoptosis. The assessment of the mitochondrial outer membrane revealed that the mice treated with the medium dose of ASP showed improved function on day 14 compared with those of the other groups (*P* < 0.05; Fig. 3c, g).

The expression of specific proteins was detected to clarify the involvement of the mitochondrial signaling pathway in AA-related apoptosis. In the AA model, the expression of Bcl-2, a primary member of the Bcl-2 family, was significantly lower compared with that in the control group, whereas the expression of the pro-apoptotic protein Bax was prominently enhanced (Fig. 3h). In addition, the Bax/Bcl-2 ratio was significantly lower in the AA group compared with the control value, and the expression levels of cleaved caspase-9 and cleaved caspase-3 in the AA group were significantly higher compared with those in the normal control group. However, the Bax/Bcl-2 ratio was significantly increased, and the expression levels of cleaved caspase-9 and cleaved caspase-3 were significantly decreased, after treatment with 200 mg/kg/d ASP (Fig. 3h). These findings indicated that ASP relieved AA apoptosis through a mitochondrion-mediated mechanism that involves Bcl-2, Bax, caspase-9, and caspase-3.

### Regulation of the abnormal apoptosis level through the p38/MAPK signaling pathway after treatment with ASP

The activation of MAPK pathways is essential for cell apoptosis, and thus, the roles of p38 MAPK pathways on AA mouse apoptosis were investigated through Western blot analysis. As shown in Fig. 3i, the medium-dose ASP treatment significantly inhibited p38 phosphorylation. These data suggested that ASP suppressed apoptosis through a mechanism associated with the inactivation of p38 pathways.

### Evalution of BMNCs and Treg cells after treatment with ASP in vitro

As shown in Fig. 4a and b, the cell viability of the model control group was significantly lower than that in the treated groups (200 ng and 400 ng) at 48 h (*P* < 0.01). Furthermore, there was no difference between 200 ng/ml and 400 ng/ml groups in the recovery of the BMNC and Treg cell levels, which indicated that 200 ng/ml is the optimal dose.

**Fig. 4:** Effects of ASP on BMNCs and Treg cells in vitro. **a**: BMNC cell viability was tested in vitro. **b**: The viability of Treg cells was detected after treatment with ASP in vitro. **c**: Markers of mitochondrial apoptosis and the p38/MAPK signaling pathway were tested by Western blotting in vitro experiments with of BMNC cells

### Preventing apoptosis through the p38/MAPK signaling pathway in BMNCs in vitro

The PrestoBlue Assay was adopted to measure the cell viability of BMNCs. As shown in Fig. 4c, after treatment with 200 ng/ml ASP, the level of Bax/Bcl-2 ratio was significantly increased and the expression levels of cleaved caspase-9 and cleaved caspase-3 and p38 phosphorylation were significantly decreased (*P* < 0.01, Fig. 4c).

## Discussion

AA is an immune-mediated bone marrow failure syndrome, and a previous study showed that the pathophysiology of AA involves the immune destruction of HSCs attacked by Th17 cells, which is correlated with the severity of AA through the specific secretion of IL-17 [20]. Impairments in the function of CD4 + CD25 + Foxp3+ Tregs in patients with AA can suppress the effects of normal effector T cells and the production of IFNγ [21]. The combination of Th1 and Th17 expansion with decreased Th2 and Treg immunophenotype and function contribute to the hematopoietic failure induced by immune attack in the bone marrow [22]. Rapamycin, which acts as a mTOR inhibitor, can ameliorate the phenotype of the immune-mediated AA model by inhibiting abnormal mitochondrial oxidative phosphorylation [23].

Alterations in mtDNA can cause damage in mitochondrial respiratory complexes, which is the primary cause of mitochondrial disease [24–26]. In addition to their close relationship to mitochondrial disease, mtDNA mutations are closely associated with cancer, diabetes, and hematological diseases through a decrease in cellular energy and the disruption of cell signaling and apoptosis, and these relationships are similar to those observed in the normal aging process [27]. It has been hypothesized that mtDNA mutations and severe pancytopenia or reticulocytopenia are closely related [28], and erythrocyte maturation and homeostasis can be accelerated if the damaged mitochondria are cleared [29]. One study showed that protecting genomic and functional integrity in the hematopoietic system, critically depends on decreasing helix-distorting oxidative nucleotide lesions and mitochondrial dysfunction [30]. Nutritional supplements can improve weight, peripheral blood, bone marrow, and histologic parameters of AA rat models by reversing abnormal levels of mitochondrial DNA content and adenosine triphosphate content, membrane potential and oxidative stress. They can also improve the number of mitochondria in the liver/spleen/kidney/ brain, as shown in this model [31].

ASP has been used for treating anemia and bone marrow damage for many years. The ASP-iron complex not only exerts an excellent curative effect on iron deficiency anemia in rats but also supplements the blood and promotes blood circulation [32]. ASP downregulates hepcidin expression by preventing activation of Janus kinase, extracellular signal-regulated kinase, and even the sons of mothers against decapentaplegic (SMAD) pathway in rats with iron deficiency anemia (IDA) [33]. Qin found that ASP can improve proteoglycan synthesis by chondrocytes in an in vivo rat osteoarthritis model by promoting the expression of aggrecan, as observed in IL-1β-stimulated chondrocytes in vitro [34]. ASP can regulate the expression of Th1 and Th2 related cytokines, the percentage of CD4(+) T cells and CD8(+) T cells among the total spleen cells [35]. Interestingly, if the drug delivery system was changed with PLGA, the level of lymphocyte proliferation and the ratio of CD4+ to CD8+ T cells was significantly improved with ASP [36]. Based on these studies, we attempted to examine the mechanism by which ASP alleviates the hematopoietic failure induced by immune attack in AA mice. In this study, the AA mouse model was induced through a combination of 60Co γ-radiation and transplanted lymph node cells. The AA mice showed statistically significant reductions in peripheral blood leukocytes, red blood cells and PLTs (Fig. 1),severe reductions in BMNCs (Fig. 1) and abnormal immune levels (Fig. 2), which are clinical characteristics of AA. The Treg/Th17 ratios obtained in this study demonstrated that ASP improved hematopoietic function through the regulation of abnormal immunity in AA (Fig. 2). However, the AA mice treated with ASP showed a progressive increase in the number of BMNCs and better ability of LSKs to decrease the mitochondrial apoptosis ratio than those belonging to the AA group (Fig. 3a and e). Additionally, the increased mitochondrial outer and inner membrane function and decreased levels of ROS that were observed in vivo verified the antagonistic effect of ASP on mitochondrial pathway apoptosis in AA mice (Fig. 3b-d, f, g). The in vivo and in vitro results also demonstrated that ASP increased the expression of Bcl-2, decreased the expression of Bax, and inactivated the caspase-9 and caspase-3 cascades, which are markers of apoptosis (Figs. 3h, j and 4c). It has been reported that Bcl-2 family proteins can mediate mitochondria-dependent pathway apoptosis [37]. Our apoptosis data confirmed that ASP reduces apoptosis through a mitochondria-mediated pathway in mice.

## Conclusion

AA model mice and vitro experiments exhibit severe impairments in mitochondrial function caused by apoptosis. The indicators of mitochondrial apoptosis and the Treg/Th17 cell ratio in the ASP-treated group, particularly the medium-dose group, were significantly better than those in the AA group, which indicates that these impairments can be ameliorated by treatment with ASP through the regulation of immune function.

## Supplementary information

**Additional file 1.**

## Data Availability

The datasets supporting the conclusions of this article are included within the article. The datasets used and/or analyzed during the current study are available from the corresponding author on reasonable request.

## Abbreviations

ASP: Angelica sinensis polysaccharide
AA: Aplastic anemia
BMNCs: Bone marrow-nucleated cells
ROS: Reactive oxygen species
MDA: Malondialdehyde
COX: Cytochrome oxidase
MDH: Malate dehydrogenase
mtDNA: Mitochondria DNA
CFU-Es: Colony-forming unit-erythrocytes
BFU-Es: Burst-forming units-erythrocyte
MMP: Mitochondrial membrane potential
